RETRACTED

# Vision Sensor-Based Real-Time Fire Detection in Resource-Constrained IoT Environments

**DOI:** 10.1155/2021/5195508

**Published:** 2021-12-21

**Authors:** Hikmat Yar, Tanveer Hussain, Zulfiqar Ahmad Khan, Deepika Koundal, Mi Young Lee, Sung Wook Baik

**Affiliations:** ^1^Sejong University, Seoul 143-747, Republic of Korea; ^2^Department of Systemics, University of Petroleum & Energy Studies, Dehradun, India

## Abstract

Fire detection and management is very important to prevent social, ecological, and economic damages. However, achieving real-time fire detection with higher accuracy in an IoT environment is a challenging task due to limited storage, transmission, and computation resources. To overcome these challenges, early fire detection and automatic response are very significant. Therefore, we develop a novel framework based on a lightweight convolutional neural network (CNN), requiring less training time, and it is applicable over resource-constrained devices. The internal architecture of the proposed model is inspired by the block-wise VGG16 architecture with a significantly reduced number of parameters, input size, inference time, and comparatively higher accuracy for early fire detection. In the proposed model, small-size uniform convolutional filters are employed that are specifically designed to capture fine details of input fire images with a sequentially increasing number of channels to aid effective feature extraction. The proposed model is evaluated on two datasets such as a benchmark Foggia's dataset and our newly created small-scaled fire detection dataset with extremely challenging real-world images containing a high-level of diversity. Experimental results conducted on both datasets reveal the better performance of the proposed model compared to state-of-the-art in terms of accuracy, false-positive rate, model size, and running time, which indicates its robustness and feasible installation in real-world scenarios.

## 1. Introduction

Wildfire, an extremely catastrophic disaster, leads to the destruction of forests, human assets, yielding reduced soil fertility, and land resources and is a major cause of global warming. Wildfire is a devastating natural disaster, having adverse effects on living beings and the ecological environment. Living places are usually surrounded by buildings, agricultural land, and forests, where the occurrence of fire incidents can be threatening for human lives and properties. Throughout the globe, wildfires, building fires, and vehicle fires have a huge impact on global warming, the ecosystem, and the economy, resulting loss of living beings. According to World Fire Statistics Report 2018, during 1993–2016, 2.5–4.5 million structure (building) fires occurred and nearly 62,000 fire deaths were reported from 57 countries [1]. According to The National Fire Data System (NFDS), in South Korea, a total of 24,539 structure fire cases were reported, causing 250 deaths, 1,646 injuries, and direct property damage of 705,960 USD from September 2020 to September 2021 [2]. From September 2020 to September 2021, in South Korea, 78,219 vehicle fires occurred, which caused 461 deaths, 1,875 injuries, and property damage of 357,609 USD [3].

RETRACTED

In contrast to building and vehicle fires, wildfires are the most dangerous disasters that affect the life cycle of nature. There are many causes of wildfires such as rising temperatures, changing climate, lightning from clouds, sparking from falling rocks, or rubbing dry trees during summers [4]. The devastation caused by wildfires has risen over the past two decades in the United States and other countries around the globe. Since 2000, an average of 72,200 forest fires have burned round about seven million acres each year, and the number of acres has doubled since the 1990s [5]. In 2016, 1,161 people were affected by wildfires in Southern Europe which resulted in a loss of 5.5 billion USD [6]. In North America and Russia, wildfires damaged 100,000 km^2^ of vegetation land. The number of people affected by wildfires in 2016 was 158,290, the third-highest since 2006, but is far from the 1 million who suffered from forest fires in Macedonia in 2007. The California Department of Forestry and Fire Prevention reported that, in the history of California, 2018 is considered one of the worst years, and they observed 7,500 fires that burned almost 1,670,000 acres and affects more than 100 lives [6]. These alarming facts motivated the researchers to develop an effective mechanism for early fire detection and its management. For this purpose, several researchers proposed soft computing techniques to prevent fires from expanding based on conventional fire alert systems (CFAS) and visual sensors [7]. In CFAS, the researchers used different kinds of scalar sensors for fire detection such as optical sensors, flame sensors, and smoke sensors that require proximity to the fire. Scalar sensors-based systems fail in the context of providing additional information such as coverage of an area, burning degree, location, and fire size. Furthermore, these sensors demand human interactions, i.e., to visit a fire location for confirmation in case of any fire alarm. Considering such limitations, the researchers proposed different techniques based on visual sensors [7]. The vision-based systems play a vital role in fire detection, where traditional fire detection (TFD) methods and DL-based methods are used in surveillance systems for automatic monitoring of fire disasters [8–10]. These algorithms have the advantages of quick response, fewer human interventions, cost affordability, and larger coverage. However, fire detection using TFD-based methods is a challenging and time-consuming process because TFD-based methods require hand-crafted features extraction, where features engineering and selection are tedious work and require domain experts. Particularly, in TFD-based methods, early fire detection and alarm generation are also challenging due to varying lighting conditions, shadows, and low detection accuracy [7]. Considering the potentials of DL models in various domains, we employ them in our research, i.e., fire detection in surveillance videos. DL provides end-to-end feature extraction mechanism, but it requires a large amount of training data and is computationally expensive. Therefore, in this paper, we developed a lightweight (LW-CNN) model with better detection accuracy, low false alarm rates, and the potential to be deployed over resource-constrained devices (RCD). The major contributions of this research work are summarized as follows:

- Tackling the limited computational resources challenge of real-world IoT devices, we introduce a lightweight deep model, functional over RCD in real-time. The proposed model achieves better accuracy with a limited number of learning parameters, i.e., 2.01 and 0.94 million reduced parameters when compared to famous lightweight NASNetMobile and MobileNetV1 networks.
- The existing wildfire detection datasets are uniform nature, yielding limited model's generalization, whereas we collected a diverse set of samples from real-world self-recorded videos, Facebook, news channel, and YouTube videos.
- We performed different experiments over Foggia's and our newly created fire detection datasets using different baseline models such as AlexNet [11], VGG16 [12], ResNet50 [13], MobileNetV1 [14], and NASNetMobile [15]. The experimental results show that the proposed model reveals better results in terms of accuracy, false alarm rates, and time complexity as compared to SOTA models.

RETRACTED

The rest of the work is structured as follows: in Section 2, we provided a brief explanation of literature along with its merits and demerits, Section 3 explained the internal architecture of the proposed model, the details about the proposed dataset and experimental results are explained in Section 4, and lastly, we conclude the paper in Section 5 with several future directions for the research community.

## 2. Related Work

In the recent literature, several researchers show their contributions in the field of fire detection including CFAS and vision sensors-based systems. In CFAS, different environmental sensors such as smoke, temperature, and photosensitive are used for fire detection [16–21]. However, CFAS methods require close distance to the fire such as indoor environment and fail for large distance fire detection such as the outdoor environments. Furthermore, the CFAS is not capable to provide extra information about the status and burning rate of the fire. The CFAS systems require human intervention, for instance, visiting a fire location to confirm fire in case of any alarm. To cope up with these limitations, many visual sensors-based fire detection systems have been presented in the literature [22, 23].

The vision-based fire detection systems are categorized into two broad categories including TFD and DL-based methods. TFD-based methods function using digital image processing and pattern recognition techniques. For instance, Liu et al. used three different methods such as temporal, spatial, and spectral analysis to detect the fire regions in an image [24]. However, their method is based on the assumption of considering the irregular shape of fire, which is not always the case as moving objects can also change their shape. TFD methods comprise wavelet analysis and fast Fourier transform [25], fire pixel classification using rule-based generic color algorithm [26]. Furthermore, Foggia et al. applied motion analysis, shape variation, color features, and bag-of-word for fire classification [27]. Existing methods also applied gray level co-occurrence matrix and histogram of oriented gradient with SVM [28], background subtraction, and color space selection for candidate fire region extraction [29]. In the TFD-based methods, handcrafted features extraction is a very tedious and time-consuming process, and these methods failed to achieve a high-level of accuracy. The DL-based methods using closed-circuit television (CCTV) surveillance systems play a vital role for fire detection, where the automatic end-to-end features extraction process makes these models more convenient and reliable.

When compared to TFD, the DL models achieved better performance in terms of increased accuracy and reduced false alarms. For instance, Frizzi et al. proposed a customized CNN-based architecture for smoke and fire detection [30]. They utilized a very limited number of images for results evaluation and did not compare their results with any SOTA method. In 2017, Sharma et al. used two pretrained SOTA CNN models for fire detection, i.e., VGG16 and ResNet50. A CNN-based model for fire detection in a surveillance system is used for surveillance disaster management [10], where authors used pretrained AlexNet model in their framework. Besides this, they presented an intelligent mechanism for camera selection based on priority. In this research work, the main problem is the time complexity of their proposed architecture which is difficult to deploy on RCD. To overcome the time complexity and increase the performance of the model, a group of researchers extended their work and used GoogLeNet resembling neural architecture for efficient fire detection in surveillance videos [31]. They performed experiments over two benchmark datasets and achieved better accuracy as compared to SOTA methods. In the next approach, Khan et al. proposed a lightweight SqueezeNet architecture for efficient fire detection and localization in surveillance [32]. In this work, they also determined the intensity of the detectable fire and the objects under observation. Khan et al. presented an energy-efficient scheme based on a deep CNN that can efficiently detect early smoke in a foggy and normal environments [8]. Furthermore, for fire detection in uncertain environments, Khan et al. proposed lightweight deep models [14, 33] based on MobileNetV2 [34], where a lightweight DCNN without dense fully connected layers is used to make it computationally inexpensive. They reduced the size of the trained model up to 3 MB, without compromising on its performance and achieved SOTA accuracy over two benchmark datasets [14]. Aslan et al. developed deep convolutional generative adversarial neural networks for fire detection in [35] that are trained over real images and noise vectors; herein, the discriminator was trained individually using smoky images without the generator. The next approach is presented by Hashemzadeh and Zademehdi, with a robust color model for candidate fire regions detection. In their proposed work, a motion-intensity-aware technique is used for motion analysis, where the spatio-temporal features are used to differentiate the fire and non-fire regions [36]. Xu et al. presented a deep saliency network to detect the forest fire regions in an image [37]. They fused the pixel and object-level salient regions from the CNNs model to extract a smoky saliency map. Shahid and Hua presented a vision transformer-based fire detection method, where they divided an image into similar size of patches to gain a long-range relationship. They evaluated their method on two benchmark datasets following Khan et al. [31, 33] evaluation strategies; however, their method is less accurate and computationally expensive as compared to the method proposed by Khan et al. A forest fire detection system using fuzzy entropy optimized thresholding and STN-Based CNN is proposed by Reddy et al. [38], where a spatial transformer network and thresholding operation based on entropy function is used in the softmax layer for fire scene classification. In the light of current literature, several DL-based strategies are developed for fire detection and achieved convincing accuracies. However, the detection accuracy further needs to be improved with reduced false alarm rates to save lives and properties from damages. Furthermore, these models are computationally expensive and require powerful GPUs and TPUs. To overcome these concerns, in this work, we developed a LW-CNN-based model for fire detection with high detection accuracy and low false alarm rates and can be deployed over RCD.

RETRACTED

## 3. The Proposed Methodology

The proposed framework comprises data preprocessing and our model definition, where data preprocessing techniques are used to prepare data for training and testing. Furthermore, data augmentation techniques such as scaling, rotation, horizontal flip, and contrast enhancement [39] are used to generate new images from the existing ones to increase the size of training examples for superior result evaluations and better generalization. The augmented datasets are used to train different CNN models. The details of each step of the proposed framework are briefly described in the subsequent sections and visualized in Figure 1.

### 3.1. Data Preprocessing

Preprocessing refers to all the transformations on the raw data before it is fed to the proposed end-to-end LW-CNN architecture. For example, training CNN architecture on raw data will reduce the classification performance. Furthermore, we increase the input data via data augmentation to generate new images with varying orientation, position, and scale, as shown in Figures 2 and 3, which will probably lead to good classification performance [39]. In the subsequent sections, we provided further details of the data augmentation steps.

*Data Augmentation*: The huge diversity of images makes CNN architectures more robust towards challenging scenarios and the models gain better classification potentials, i.e., making it aware of all kinds of data structures with varied scaled objects and their orientations. This way, a deep model has to deal with all these variations, which is possible via data augmentation [40], that is one of the most prominent techniques to generate new images from the existing ones by applying different image transformations and enhancement techniques. During data augmentation, the model learns the same object present in the image with different perspectives which increases the generalization ability of the model. For this purpose, we employ several data augmentation and enhancement techniques before training the model.
*Geometric Transformations:* This step includes rotation, scaling, and horizontal flipping, and we have used these steps on each image in the dataset to get five more images from this transformation alone, as shown in Figure 2.
*Contrast Enhancement*: This step is used to remove the effects of contrast variations from images due to varying light conditions. The contrast stretching technique defined in equation (1) is applied on the input image to introduce contrast variations,as given in Figure 3.
In equation (1), *g*(*x*, *y*) is the output image, where *f* (*x*, *y*) is the input pixel value; *s*_1_, *s*_2_, *r*_1,_ and *r*_2_ are the contrast adjustment parameters; *a*_1_, *a*_2_, and *a*_3_ are scaling factors for various grayscale regions.
  (1) $$\begin{array}{c} g\left(x,y\right)=\left\{\begin{array}{c} a_{1}f\left(x,y\right)f\left(x,y\right)<r_{1}\\ a_{2}\left(f\left(x,y\right)-r_{1}\right)+s_{1},r_{1}\geq f\left(x,y\right)<r_{2}\\ a_{3}\left(f\left(x,y\right)-r_{2}\right)+s_{2},f\left(x,y\right)<r_{2} \end{array}\right\}. \end{array}$$

RETRACTED

### 3.2. The Proposed Model Description

CNNs are widely used and in complex visual recognition tasks such as action and activity recognition [41], anomaly detection and recognition [42, 43], classification [44, 45], object detection [46], and a variety of other recognition, video summarization, and segmentation tasks [41–49]. The CNN architecture consists of convolutional layers (CL), pooling layers, and fully connected layers. Deep CNN consists of a single input, several hidden, fully connected, and softmax layers. In deep CNN, there are several numbers of parameters, local receptive fields, and different kernels that are used to generate feature maps to extract prominent features from the objects present in the image. These feature maps are mostly subsampled by using average, min, or maxpooling for dimensionality reduction. The selection of a suitable CNN model for a particular problem is also a challenging task to acquire accurate predictions and balance them with the computational complexity. To this end, we first analyzed the performance of well-known ImageNet [50] and pretrained CNN architectures such as AlexNet, VGG16, ResNet50, MobileNetV1, and NASNetMobile, before introducing our newly created LW-CNN model. Our model is specifically designed to capture fire regions effectively from visual data. Therefore, we process a reduced size of the input image, which unlike existing CNNs [12], captures fire regions effectively. Furthermore, small-sized uniform filters are deployed in our model to capture every type of small detail from an input image, generating more representative features for classifier learning.

 
*Implementation details*: In the context of architecture setup, each CNN has its own merits and demerits such as the designing and development of AlexNet and VGG16 architectures are easy to implement, where AlexNet architecture is considered as the baseline architecture in DL, first appeared in the ImageNet contest and achieved astonishing results [11]. The VGG explores the impact of increasing the number of CL in the network to improve its performance. The authors proposed VGG16, a 16-layered architecture with the same filter size, which is a robust feature extractor and performs better on large-scale datasets and complex background recognition tasks and shows significant improvement in the classification task. Despite the several advantages of AlexNet and VGG16, these architectures are computationally expensive in terms of model size and learning parameters. The NASNetMobile, MobileNetV1, and ResNet50 are the recent, robust, and computationally less-expensive CNN architectures, where MobileNetV1 and NASNetMobile are specifically designed for RCD. Considering the motivation of RCD resources and overcoming the limitations of existing lightweight models, we designed our CNN architecture, which is more suitable for RCD because of its time complexity and trustworthy results for the task under investigation. A significant reduction is found in the learning parameters while comparing the proposed model with famous lightweight NASNetMobile and MobileNetV1 networks. The proposed LW-CNN learns 3.31 million parameters during training, which are 2.01 and 0.94 million fewer parameters than NASNetMobile and MobileNetV1, respectively. The proposed LW-CNN model includes an input layer, three CL, two fully connected layers, and one softmax layer. Each CL is followed by a batch-normalization and subsampling layer (maximum pooling). In the first CL, the input image is 128 × 128 having three channels: red, green, and blue with 32 different filters for deep features extraction, the size of each filter is 3 × 3, and we set a 1-pixel stride. In the second and third CL, the number of filters is increased to 64 and 128, respectively, and the remaining parameters are similar to the ones in the first CL. In the proposed model, we used the ReLu activation function in each layer. Next, in the first and second fully connected layer, 128 and 64 neurons are selected based on different experiments, and the output is fed into a softmax layer which produces a distribution over the two class labels such as fire and non-fire. The training parameters of the proposed model are given in Table 1.

RETRACTED

## 4. Results and Discussion

This section provides a detailed discussion about, evaluation metrics, datasets, and visual results. Firstly, we explained experimental setup and performance metrics, next we provided dataset explanation, and finally presented results evaluation.

 
*Training Details*. All the models (ablation study) including ours are trained using 30 epochs with a small learning rate so that most of the previously acquired knowledge can be retained in the network. The pretrained model moderately updates the learning parameters for achieving optimal results on the target dataset. The various hyperparameters used in our ablation experiments are presented in Table 2. Thus, we used the default input size of each network to retrain with a batch size of 32, and the stochastic gradient descent optimizer with momentum (SGD-M) set to 1*e*-4 with 0.9 momentum.
  The experiments are performed on NVIDIA GTX 2060 Graphics Processing Unit (GPU) with 16 Gigabyte (GB) onboard memory using the Keras DL framework with TensorFlow backend. The performance of the proposed model is evaluated on several evaluation matrices such as accuracy, precision, recall, F1-measure, false-negative rate (FNR), and false-positive rate (FPR) (also referred to as false alarm rate) [32], as stated in the following equations:

(2) $$\begin{array}{c} \text{accuracy}=\left(\frac{\text{TP}+\text{TN}}{\text{TP}+\text{TN}+\text{FP}+\text{FN}}\right), \end{array}$$

(3) $$\begin{array}{c} \text{precision}=\;\left(\frac{\text{TP}}{\text{TP}+\text{FP}}\right), \end{array}$$

(4) $$\begin{array}{c} \text{recall}=\left(\frac{\text{TP}}{\text{TP}+\text{FN}}\right), \end{array}$$

(5) $$\begin{array}{c} \text{F}1-\text{score}=2*\left(\frac{\text{precision}*\text{recall}}{\text{precision}+\text{recall}}\right), \end{array}$$

(6) $$\begin{array}{c} \text{FPR}=\left(\frac{\text{FP}}{\text{FP}+\text{TN}}\right), \end{array}$$

(7) $$\begin{array}{c} \text{FNR}=\left(\frac{\text{FN}}{\text{TP}+\text{FN}}\right)\text{.} \end{array}$$

### 4.1. Datasets and Result Evaluation

In this section, we briefly explained the datasets used in this work such as Foggia's video dataset [27] and our newly created fire detection dataset. We performed different experiments with various CNN models to evaluate the performance of the proposed work.

#### 4.1.1. Results Evaluation Using Foggia's Dataset

We selected Foggia's dataset to evaluate and compare the performance of the proposed LW-CNN architecture with SOTA methods. Foggia's dataset is a widely used publicly available benchmark dataset consisting of 31 videos of indoor and outdoor environments, where 14 videos contain fire scenes, and the remaining are related to non-fire scenes. A total of 14,036 images are obtained from these videos, which are then equally distributed to both classes such as fire and non-fire, and each class consists of 7,018 images. We used 70% images for training, 20% for validation, and the remaining 10% are used for testing. The sample images of Foggia's dataset are shown in Figure 4. The accuracy and loss graph of the proposed model over Foggia's dataset is shown in Figure 5. In the experiments, the model is trained over 30 epochs using an SGD optimizer. The training and validation accuracy is presented in Figure 5(a), where Figure 5(b) represents training and validation loss. As shown in Figure 5, the training and validation accuracy is gradually increasing after each epoch. On the 15^th^ epoch, the model is converged with 99% training and 97% validation accuracy.

RETRACTED

The classification report of the proposed model over test data is given in Table 3, where the precision, recall, and F1-score of fire class are 0.97, 0.98, and 0.97, respectively, and the precision, recall, and F1-score of non-fire class are 0.96, 0.97, and 0.96, respectively.

The confusion matrix of the proposed model over test data using Foggia's dataset is shown in Figure 6, where the intensity of true positives is high for both categories; the proposed model achieved 99% and 96% accuracy for fire and non-fire class, respectively, which proves the efficiency of the proposed model over Foggia's dataset.

The performance of the proposed model is compared with ANetFire [7], GNetFire [31], CNNFire [32], ICA_K [36], ViT-B/32 [51], and STN-CNN [38]. The experimental results from Foggia's dataset in terms of FPR, FNR, and accuracy are given in Table 4. We can observe that ANetFire scored FPR of 9.07 and FNR of 2.13 with an accuracy of 94.39%. The FPR, FNR, and accuracy achieved by GNetFire are 0.054, 1.5, and 94.43%, respectively. The CNNFire achieved FPR of 8.87, FNR of 2.12, with accuracy of 94.50%. Similarly, ICA_K obtained 4.83, 4.53, and 95.32% FPR, FNR, and accuracy, respectively. The STN-CNN achieved an accuracy of 96.23%, where the FPR and FNR is 3.68 and 2.46, respectively. The FPR, FNR, and accuracy of ViT-B/32 are 2.15, 1.02, and 94.03%, respectively. Our proposed model overwhelmed the SOTA techniques and achieved lowest false alarming rates and highest accuracies such as 0, 0.92, and 97.15% FPR, FNR, and accuracy, respectively.

The dataset provided by Foggia et al. [27] consists of 31 fire and non-fire videos, the dataset is vast, and it is not diverse enough to be used completely to train a network for real-world scenarios, where many deep models can achieve higher training and testing accuracy, but fail in generalizing their predictions [52]. The reason behind their restricted generalization is the limited diversity of this dataset, as it contains a large number of similar images that are extracted from videos with a smaller number of frames skip among consecutive frames, producing almost similar images for training and testing. Therefore, we develop a diverse dataset for forest fire detection. Although the dataset may appear to be small, it is extremely diverse; a detailed explanation is given in Section 4.1.2.

RETRACTED

#### 4.1.2. Result Evaluation Using the Proposed Dataset

The experiments are performed on the newly created dataset, which includes forest fire and non-fire classes with a total number of 2,000 images, and each class consists of 1,000 images. The fire images are collected from different sources, i.e., real-world self-recorded videos, Facebook, news channel, and YouTube videos. The source- and country-wise percentages of collected data are given in Figure 7, and the information about the length of the video and its corresponding extracted frames is given in Table 5. For the non-fire class, we selected 107 non-fire images from Bowfire datasets [53]. It is a small dataset consisting of two fire and non-fire classes, the total number of images in the Bowfire dataset is 226, where the fire class consists of 119 images while the rest of the images belong to the non-fire class. Instead of the BowFire dataset, we collected 893 images from Google, the non-fire class is extremely challenging for the model to train such as fire-colored lighting, fire-like sunlight, and fire-colored objects in different buildings. Our codes and datasets are available at https://github.com/Hikmat-Yar.

Furthermore, the dataset is divided into three subgroups, i.e., training, validation, and testing, and the training set consists of 70% of the total dataset, where 20% is used for validation and the remaining 10% is considered for testing. Some sample images of the proposed dataset are given in Figure 8. The classification report of the proposed model over a custom dataset is given in Table 6, and its comparison with the SOTA CNN models is given in Table 7, where the training accuracy and loss graph are shown in Figure 9. During experiments, we trained each model for 30 epochs, and the proposed model achieved the highest accuracy compared to other models. A detailed analysis of each model can be extracted from the confusion matrix as depicted in Figure 10. The blue diagonal corresponds to the true positives, where the saturation indicates the accurate classification.

The proposed model provided good classification results as compared to other models and accurately classified as fire and non-fire images. Some of the samples in both categories were misclassified, i.e., forest fire as non-fire and vice versa. It is understandable to keep in view the visual similarities in both these categories.

RETRACTED

The accuracy and loss graph of the proposed model is visualized in Figure 9. The horizontal axis represents the number of epochs, and the vertical axis shows accuracy and loss.

In Figure 9, it can be observed that the proposed model performs well for forest fire detection. During the training and validation of the model, as the number of iterations increases, the model accuracy and loss values change, as shown in Figure 9(a). The proposed model is converged on 28 epochs, where training and validation accuracy reached 98% and 96%, respectively. Similarly, the training and validation loss of the proposed model reached 0.1 and 0.22, respectively, as depicted in Figure 9(b).

Figure 10 shows the confusion matrix of each model on the proposed dataset, where Figure 10(a) represents AlexNet, Figure 10(b) represents ResNet50, Figure 10(c) represents NASNetMobile, Figure 10(d) represents MobileNetV1, Figure 10(e) represents VGG16, and Figure 10(f) represents the proposed model. In the experiments, the correct prediction of the model Figure 10(a) for fire and non-fire class is 0.93 and 0.78, respectively, where the misclassification is 0.07 and 0.22, respectively. Similarly, the correct prediction of models Figures 10(b)–10(d) and Figure 10(e) for fire class are 0.96, 0.95, 0.99, and 0.93, respectively; for non-fire class, the correct prediction of these models is 0.77, 0.88, 0.86, and 0.94, respectively. The proposed model is represented by Figure 10(f), where the correct prediction of fire and non-fire class is 0.98 and 0.91, respectively. The misclassification of the model Figure 10(f) for the fire and non-fire class is 0.02 and 0.09, respectively. Therefore, the confusion matrix of all these models confirms that the proposed model dominated all the mentioned models in our experiments.

The classification report of the proposed model over the proposed dataset is given in Table 6, where the precision, recall, and F1-score of the forest fire (positive) class and non-fire (negative) class are measured. Our proposed model for forest fire achieved precision, recall, and F1-scores of 0.91, 0.98, and 0.95, respectively, and for non-fire, the proposed model achieved precision, recall, and F1-scores of 0.98, 0.91, and 0.94, respectively.

The comparison of the proposed model with other baseline-CNN models using FPR, FNR, and accuracy is given in Table 7, where AlexNet and ResNet50 models encountered overfitting and achieved the worst results in terms of FPR, FNR, and accuracy, while the proposed model attains 9% and 7.83% higher accuracy from the AlexNet and ResNet50 models, respectively. To compare with NASNetMobile, the FPR and FNR of the NASNetMobile are 4 and 12, while achieving 3% less accuracy than the proposed model. Furthermore, to compare with MobileNetV1, the FPR of the proposed model is similar to MobileNetV1. However, the proposed model achieved 2.1% higher accuracy than the MobileNetV1 with 7 FNR value. The proposed model achieved good results than the heavier VGG16 model due to the relatively smaller dataset being insufficient to tune the extremely large number of parameters. The results of the VGG16 are close to the proposed model; in the case of FNR, the VGG16 model achieved lower FNR but its FPR is high and achieved 1.33% fewer accuracy against the proposed model. In the experiments, the AlexNet and ResNet50 model introduced overfitting after 19 and 22 epochs, respectively, where the NASNetMobile, MobileNetV1, and VGG16 are converged on 21, 24, and 26 epochs, respectively, whereas, in Figure 9, it can be seen that the proposed model is converged on 28 epochs.

RETRACTED

From Table 7, it is observable that, the AlexNet model achieved 85.50% accuracy which is the lowest in our experiments, the VGG16 and proposed model achieved 93.17% and 94.50%, respectively, which are the highest accuracies, but the VGG16 model is not suitable for RCD due to model size and processing time. The proposed model achieved good results in terms of accuracy, FPR, and FNR and is more suitable for RCD. The proposed model is functional over RCD in almost real-time, where uniform convolutional filters employed in our network are specifically designed to capture fine details of input fire images with a sequentially increasing number of channels to aid effective feature extraction. The better accuracy, FPR, and FNR rates obtained by the proposed model confirm that the small and uniformity in the filter size extract rich features to train the model.

### 4.2. Time Complexity Analysis

To evaluate a model's efficiency, it is important to check its performance and deployability potentials in real-time over different devices such as GPU, CPU, and RCD. The specification of GPU and CPU are given in training details in Section 4, and RCD used in our experiments is Raspberry Pi 4 (RPI). It is a Broadcom BCM2711, Quad-core Cortex-A72 (ARM v8) 64-bit SoC @ 1.5 GHz system, having 4 GB of SDRAM. Considering these three different setups, we examine the frame per second (FPS) of our proposed model, where the FPS of the proposed model using GPU, CPU, and RPI is 200.35, 21.02, and 16.02 FPS, respectively. The comparison of our proposed work in terms of FPS with different baseline models is given in Table 8.

RETRACTED

In our experiments, the FPS of the AlexNet model using GPU, CPU, and RPi is 95.22, 4.88, and 0.90, respectively. The FPS of the original VGG16 model is 78.06, 2.96, and 0.60 respectively, The ResNet50 model has 101.31, 6.35, and 1.07 FPS, respectively. The NASNetMobile model gives 110.57, 12.76, and 3.24 FPS, respectively, while the MobileNetV1 model process 130.88, 15.47, and 9.05, respectively. The time complexity of the proposed model is better as compared to other baseline models, so the proposed model is applicable for real-time implementation over RCD. Besides this, we can use Intel Movidius Neural Compute Stick to increase the FPS of our proposed work. The Neural Compute Stick is a small, USB-based low-powered coprocessor that is used in the deployment of different CNN models over RCD. The NCS is powered by the Myriad2 Vision Processing Unit (VPU) and supports C++ or Python API [54]. During inference, the VPU shows 40 times faster performance than RPI 3 [55]. Furthermore, the visualized results of the proposed model can be seen in Figure 11.

## 5. Conclusion

In early fire scene classification using a smart surveillance system, CNN plays a vital role to prevent social, ecological, and economic damages. However, the current literature focuses to improve the accuracy of fire detection without considering the computational cost and generalization abilities in real-world scenarios. Therefore, we proposed a LW-CNN architecture that can be deployed over RCD to utilize the embedded capability of RCD for fire detection. Inspired by the small size uniform convolutional filters of VGG16, we designed a LW-CNN architecture having three convolution layers, two dense layers, and a softmax layer where a small size uniform convolutional filter with a sequentially increasing number of channels is used to extract fine details from an input image. The proposed model is evaluated on two datasets such as a benchmark “Foggia's” dataset and our newly created fire dataset for experimental evaluations. The proposed model achieved 1.33% higher accuracy over the SOTA baseline CNN models on the proposed dataset and boosted the SOTA accuracy up to 1.83% on Foggia's dataset. The FNR and FPR of the LW-CNN model on the proposed dataset are 1.2 and 7 and on Foggia's dataset are 0 and 0.92, respectively. The proposed model reveals good results in terms of accuracy, false alarm rates, and running time for the considered datasets. Additionally, we achieved 200.35, 21.02, and 16.02 FPS over GPU, CPU, and RCD, respectively, indicating the robustness and feasible installation of the proposed model in a smart surveillance system

The proposed system consists of a few convolution layers, which reduces the computational complexity and are well suited for RCD. However, this system can overfit while increasing the number of classes in the dataset and can fail in an uncertain environment having fog, haze, snow, etc. Furthermore, the FNR and FPR of the proposed model are still high for our newly created dataset due to the huge diversity in our dataset and the high-level of visual similarity between fire and non-fire images.

RETRACTED

In the future, we aim to use pruning and quantization techniques to make the proposed model more efficient with a reduced number of learning parameters and model size that are more effectively deployable over RCD with online learning abilities for non-stationary environments. We also aim to reduce the FNR and extend the proposed dataset further by adding new images having fog, snow, haze, etc. and adding new classes which clearly identify the objects under the fire such as vehicle fire, building fire, forest fire, and electric pole fire.

## Figures and Tables

**Figure 1:** The proposed framework for fire detection with data preprocessing, testing procedure, and the proposed model detailed definition.

**Figure 2:** Actual and generated images of geometric transformations to increase the number of samples in the dataset, where (a) represents an original image; (b) represents horizontal flip; (c) represents scaling; (d, e, f) represent rotation with different degrees.

**Figure 3:** Different stages of contrast enhancement, where (a) represents low-contrast, (b) medium, and (c) high contrast.

**Figure 4:** Sample images of Foggia's dataset, where (a) represents fire and (b) represents non-fire images.

**Figure 5:** (a) Training and validation accuracy, (b) training and validation loss.

**Figure 6:** Confusion matrix of the proposed model over Foggia's dataset, where the predictions in the figure are normalized between zero and one.

**Figure 7:** Overall distribution of collected data. (a) Percentage of country-wise collected data and (b) represents sources from which the data is collected.

**Figure 8:** Sample images of the proposed dataset: (a) fire and (b) non-fire images of the dataset.

**Figure 9:** Training and validation loss and accuracy of the proposed model, where it can be observed that, in (a), the accuracy after 30 epochs converged, and similarly, in (b), the loss becomes constant after 27 epochs, indicating that the model has reached its learning limits.

**Figure 10:** The confusion matrix of each model. (a) AlexNet, (b) ResNet50, (c) NASNetMobile, (d) MobileNetV1, (e) VGG16, and (f) the proposed LW-CNN model.

**Figure 11:** The visualized results of the proposed model for early fire detection in the real-time scenario (a) represents non-fire and (b) represents forest-fire images.

RETRACTED

**Table 1:** Network training parameters.

Layer (type)	#Filter	Kernel size	Stride	#Param (million)
Convolution 1	32	(3, 3)	1	0.000896
Activation (ReLu)	—	—	—	—
Batch normalization	—		—	0.000128
Maxpooling	—	(2, 2)	1	—
Convolution 2	64	(3, 3)	1	0.018496
Activation (ReLu)	—	—	—	—
Batch normalization	—		—	0.000256
Maxpooling	—	(2, 2)	1	—
Convolution 3	128	(3, 3)	1	0.073856
Activation (ReLu)	—	—	—	—
Batch normalization	—		—	0.000512
Maxpooling	—	(2, 2)	1	—
Dropout (0.2)	—	—	—	—
Flatten	—	—	—	—
Dropout (0.2)	—	—	—	—
Dense (128)	—	—	—	3.21
Dense (64)	—	—	—	0.008256
Softmax (2)	—	—	—	0.000130
Total params				3.31

**Table 2:** Input size and network training parameters of different CNN models.

Architecture	Input size	Batch size	Learning rate	Parameters (million)
AlexNet	227 × 227	32	1*e* − 4	60
VGG16	224 × 224	32	1*e* − 4	138.35
Resnt50	224 × 224	32	1*e* − 4	25.63
MobileNetV1	224 × 224	32	1*e* − 4	4.25
NASNetMobile	224 × 224	32	1*e* − 4	5.32
The proposed model	128 × 128	32	1*e* − 4	3.31

**Table 3:** Classification report of the proposed model over Foggia's dataset.

Class	Precision	Recall	F1-score
Fire	0.97	0.98	0.97
Non-fire	0.96	0.97	0.96

**Table 4:** Comparison of the proposed model with other SOTA models over Foggia's dataset.

Technique	FPR	FNR	Accuracy (%)
ANetFire [7]	9.07	2.13	94.39
GNetFire [31]	0.054	1.5	94.43
CNNFire [32]	8.87	2.12	94.50
ICA_K [36]	4.83	4.53	95.32
STN-CNN [38]	3.68	2.46	96.23
ViT-B/32 [51]	2.15	1.02	94.03
The proposed model	**0**	**0.92**	**97.15**

The best performance is shown in bold.

**Table 5:** Length and extracted frames of each video.

Video	Length (sec)	Frames	Video	Length (sec)	Frames
1	29	7	17	220	7
2	20	24	18	27	14
3	21	24	19	75	16
4	126	102	20	187	46
5	31	11	21	108	31
6	41	23	22	15	11
7	46	19	23	1389	130
8	101	47	24	1204	58
9	15	8	25	244	38
10	13	6	26	72	19
11	14	14	27	176	5
12	20	5	28	81	35
13	142	18	29	132	8
14	287	114	30	111	29
15	95	15	31	238	26
16	303	90			

**Table 6:** Classification report of forest fire and non-fire using different CNN models using the proposed dataset.

Methods	Forest fire			Non-fire		
	Precision	Recall	F1-score	Precision	Recall	F1-score
AlexNet	0.83	0.93	0.86	0.91	0.79	0.85
ResNet50	0.82	0.96	0.87	0.95	0.77	0.86
NASNetMobile	0.90	0.95	0.92	0.94	0.88	0.91
MobileNetV1	0.87	**0.99**	0.93	0.98	0.86	0.92
VGG16	**0.94**	0.93	0.93	0.92	**0.94**	0.93
The proposed model	0.91	0.98	**0.95**	**0.98**	0.91	**0.94**

The best performance is shown in bold.

**Table 7:** Performance of different DL-based models for fire detection using the proposed dataset.

Technique	FPR	FNR	Accuracy (%)
AlexNet	6	21	85.50
ResNet50	3	23	86.67
NASNetMobile	4	12	91.50
MobileNetV1	**1.20**	14	92.40
VGG16	7	**6**	93.17
The proposed model	**1.20**	7	**94.50**

Best performance is shown in bold.

RETRACTED

**Table 8:** The time complexity of different pretrained CNN models using GPU, CPU, and RPi.

Method	FPS		
	GPU	CPU	RPi
AlexNet	95.22	4.88	0.90
VGG16	78.06	2.96	0.60
ResNet50	101.31	6.35	1.07
NASNetMobile	110.57	12.76	3.24
MobileNetV1	130.88	15.47	9.05
The proposed model	**200.35**	**21.02**	**16.02**

The best performance is shown in bold.

## Data Availability

The data and related material (codes and implementation) can be found at https://github.com/Hikmat-Yar.
